The article "Evaluation of antioxidant activities, toxicity studies and the DNA damage protective effect of various solvent extracts of Litsea cubeba fruits" was retracted in 2024. Reasons: suspected computer-generated content; unreliable results or conclusions.

# Evaluation of antioxidant activities, toxicity studies and the DNA damage protective effect of various solvent extracts of *Litsea cubeba* fruits

**DOI:** 10.1016/j.heliyon.2020.e03637

**Published:** 2020-03-25

**Authors:** Tapan Seal, Kausik Chaudhuri, Basundhara Pillai, Shrabana Chakrabarti, Tanmoy Mondal, Biswajit Auddy

**Affiliations:** a Plant Chemistry Department, Botanical Survey of India, Howrah, India; b Chigurupati Technologies Private Limited, Hyderabad, India; c West Bengal University of Technology, Kolkata, India

**Keywords:** Food science, Antioxidant activity, Effect of solvent, DNA protective, *Litsea cubeba*, Toxicity

## Abstract

*Litsea cubeba* is devoured by the ethnic individuals of Arunachal Pradesh in India as food and has been traditionally used for curing different ailments. The purpose of present study was to investigate the antioxidant activities of fruits of *L. cubeba* using different solvent extracts, quantification of phenolics, toxicity studies and DNA damage protective activities. The antioxidant activities of fruits using five different solvent extracts completed utilizing different *in vitro* examines. The quantitation of phenolic and polyphenolic compounds in the methanol extract of the fruits was carried out by HPLC. The *in vitro* haemolytic examination of plant concentrates were completed on rat erythrocytes. Appraisal of cytotoxicity of eatable fruits was assessed by MTT measure. The genotoxicity of the contemplated plant was tried by the single-cell gel electrophoresis comet measure. The DNA defensive impacts of the aqueous extracts of fruits on rodent lymphocyte DNA lesions were likewise assessed with the comet test. The extract obtained by methanol exhibited the highest antioxidant activity. The HPLC examination of the methanol concentrate of the plant demonstrated the occurrence of different phenolic acids and flavonoids like caffeic acid (145.96μg/100mg DE), syringic acid (125.85 μg/100mg DE), ferulic acid (155.89 μg/100mg DE), apigenin (28.43 μg/100mg DE), kaempferol (53.41 μg/100mg DE) etc. in various amounts. The consequences of haemolytic lethality, cytotoxicity and genotoxicity of fluid concentrates of the edible plant ensure the security at cell and genomic level. The fluid concentrate of the plant fundamentally repressed DNA harm and these information recommend that the watery concentrate of *L. cubeba* can forestall oxidative DNA harm to rodent lymphocytes, which is likely because of antioxidant constituents in the concentrate. These outcomes demonstrate that *L. cubeba* can be utilized in dietary applications with a possibility to diminish oxidative pressure.

## 1 Introduction

Oxidation is a chemical reaction including the loss of electrons which can deliver free radicals. Antioxidants are synthetic or natural substances that may hinder the oxidation of different atoms. As cell reinforcements have been represented to turn away oxidative mischief realized by free radical, it can interfere with the oxidation technique by reacting with free radicals, chelating reactant metals and besides by going about as oxygen scroungers [1]. Reactive oxygen species (ROS) impact alive cells and these radicals are in charge of numerous endless illnesses in individual, for example, atherosclerosis, parkinson's malady, joint pain, alzheimer's sickness, stroke, unending fiery ailments, malignant growths, and other degenerative ailments [2]. Plant materials are rich wellsprings of active ingredients of fluctuated synthetic attributes. Concentrates on herbal plants, vegetables, and fruits have revealed the immediacy of dynamic segments *viz*. phenolic compounds, flavones, isoflavones, flavonoids, anthocyanin, coumarin, lignans, catechins and isocatechins and they have been represented to have various natural impacts, including cancer prevention agent activity [3]. Cell reinforcements from plant materials end the activity of free radicals therefore protecting the human being from various infirmities.

The article "Evaluation of antioxidant activities, toxicity studies and the DNA damage protective effect of various solvent extracts of Litsea cubeba fruits" was retracted in 2024. Reasons: suspected computer-generated content; unreliable results or conclusions.

The cell reinforcement exercises of plants are firmly dependant on the polarity of the solvents and plant parts utilized for the all-out extraction of active constituents [4, 5]. Solvents, for example, methanol, ethanol, acetone, chloroform, ethyl acetic acid derivation and water have been broadly utilized for the extraction of cell reinforcement mixes from different plants and plant based sustenances and drugs.

*Litsea cubeba* Pers., Lauraceae is overwhelming in tropical and subtropical areas of India, China, Taiwan, and Japan. The plant has therapeutic properties and has been customarily utilized for re-establishing diverse gastro-intestinal infections alongside diabetes, edema, cold, joint pain and asthma. The fruit of the plant is used in decoction for the treatment of vertigo, paralysis. The Fruits are sold in the markets in Arunachal Pradesh, India to be eaten raw or as pickles due to their carminative properties [6].

As of late, analysts have looked to separate ground-breaking and nontoxic regular cell reinforcements from consumable plants not exclusively to avert autoxidation and lipid peroxidation, yet in addition to supplant manufactured cancer prevention agents. The fruits of *L. cubeba* has been more regularly utilized as a sustenance than for restorative reason, which pulled in our interest to explore the antioxidant action of the fruit. Since out of date events plants have been used as sustenance and solutions and it is moreover understood that, when in doubt, green plants are a basic wellspring of antimutagens similarly as standard perilous masters [7]. So it is essential to choose if the wild plants can convey adversarial impacts on living being before usage. Various examinations have exhibited that plant-inferred natural compounds show defensive exercises against genotoxicity brought about by oxidative stress [8], and there is specific enthusiasm for common substances distinguished from herbal compounds. To our knowledge, there is no report in the writing on the cell reinforcement capability of *L. cubeba* fruits in various dissolvable framework. The primary objectives of this investigation were to investigate the antioxidant activities of *L. cubeba* fruits in five different solvent extracts, quantification of phenolics and flavonoids by HPLC, toxicity studies and protective effects on hydrogen peroxide (H_2_O_2_) induced DNA damage in rodent lymphocytes by comet analyse.

The article "Evaluation of antioxidant activities, toxicity studies and the DNA damage protective effect of various solvent extracts of Litsea cubeba fruits" was retracted in 2024. Reasons: suspected computer-generated content; unreliable results or conclusions.

## 2 Materials and methods

### 2.1 Plant materials

The fresh fruits of *Litsea cubeba* were gathered from Arunachal Pradesh state, India and identification was verified in our office. The voucher specimens were preserved in the Plant Chemistry Department. The edible parts were shed-dried, crushed and stored in an airtight container for further extraction.

#### 2.1.1 Chemicals and equipments

The standard phenolic and polyphenolic compounds e.g. (gallic acid, protocatechuic acid, catechin, rutin, gentisic acid, vanillic acid, caffeic acid, syringic acid, *p*-coumaric acid, ferulic acid, sinapic acid, salicylic acid, chlorogenic acid, *p-*hydroxy benzoic acid, ellagic acid, myricetin, quercetin, naringin, apigenin and kaempferol), ABTS,2′-azino-bis(3-ethylbenzothiazoline-6-sulfonicacid), DPPH (1, 1-Diphenyl-2-picrylhydrazyl), MTT (3-(4,5-Dimethylthiazol-2-yl)-2,5-Diphenyltetrazolium Bromide) were purchased from Sigma Chemical Co. (St. Louis, MO, USA). The other chemicals like, Hank's Balanced Salt Solutions (HBSS), Roswell Park Memorial Institute (RPMI), Fetal bovine serum (FBS); Dimethyl sulfoxide (DMSO), Low melting point agarose (LMPA), Normal melting point agarose (NMPA), Folin-Ciocalteus's phenol reagent, potassium ferricyanide, potassium per sulphate, Aluminium chloride, FeCl_3_, sodium carbonate, Sodium dihydrogen phosphate and trifluoroacetic acid and the HPLC-grade solvents such as acetonitrile, methanol, water, were purchased from Merck (Germany). All the chemicals used including the solvents, were of analytical grade.

HPLC analysis were achieved using Dionex Ultimate 3000 liquid chromatograph attached with a diode array detector (DAD) with 5 cm flow cell. Chromeleon system manager was used as data processor. The separation was achieved by a reversed-phase Acclaim C18 column (5 micron particle size, 250 × 4.6 mm). Fluorescence microscope (Leica Upright Fluorescence Microscope Model DM2000 with Digital Photography attachment) was used for the comet assay study.

The article "Evaluation of antioxidant activities, toxicity studies and the DNA damage protective effect of various solvent extracts of Litsea cubeba fruits" was retracted in 2024. Reasons: suspected computer-generated content; unreliable results or conclusions.

### 2.2 Antioxidant activities determination of *L. cubeba* in different solvent extracts

#### 2.2.1 Extraction of plant material

Fresh fruits of *Litsea cubeba* were collected from Itanagar, Arunachal Pradesh, washed meticulously with tap water and then with distilled water. The fruits were dried at room temperature and pulverized in a grinder machine and stored in an air-tight container. One hundred gram (100g) powdered fruits of *L. cubeba* was soaked twice in water with constant stirring for 24 h at room temperature and filtered to get the water extract. Concentrates acquired from the first and the subsequent extractions were combined and concentrated using a rotary evaporator under reduced pressure to obtain viscous extracts which were further dried using a freeze drier. Additionally, the convention was repeated with methanol, acetone, chloroform and benzene. The dry extracts were stored at -20 °C until use. The dry extract obtained with each solvent was weighed. The percentage yield was expressed in terms of air dried weight of plant material.

#### 2.2.2 Antioxidant activities determination of *L. cubeba*

The Folin-Ciocalteu method was adopted to resolve the total phenolic content (TPC) of the diverse plant concentrates and it was expressed as gallic acid equivalent (GAE) in mg/100g dry extract of concentrate (DE) [9]. The total flavonoids substance was evaluated as Rutin equivalent (RE) mg/100g dry extract of plant [9]. The reducing power capacity of the concentrates was determined as ascorbic acid identical (AAE) in mg/100g of dry concentrate [9]. Ferric reducing antioxidant power (FRAP) test was completed utilizing the technique described by Datta et al. 2019 [9] and antioxidant capacity was determined as Trolox equivalent (TE) in mg/100g dry concentrate. The free radical scavenging activity of the plant extracts was carried out utilizing the stable radical DPPH (1,1-diphenyl-2-picrylhydrazyl) [9]. The 2,2′-azino-bis(3-ethylbenzothiazoline-6-sulfonic acid) (ABTS) radical cation (ABTS.+) scavenging activity was estimated by the procedure defined by Datta et al. 2019 [9]. The metal chelating action and anti-lipid peroxidation was eavaluated following the strategy undertaken by Datta et al. 2019 [9].

### 2.3 Estimation of phenolic acids and flavonoids in *L. cubeba* by HPLC

The chromatographic investigation was done following the method as described by Datta et al. (Datta et al., 2019). The method was validated according to the USP and ICH guidelines. 20 mg dry methanol extract of *L. cubeba* dissolved in 20 ml mobile phase solvent (methanol: 0.5% acetic acid in water: 1:9) and the sample solution was filtered through 0.45 *μ*m membrane filter before injection into HPLC system. The HPLC analysis was carried out using the mobile solvent phase containing methanol (Solvent A) and 0.5% aq. acetic acid solution (Solvent B). The column was thermostatically controlled at 25 °C and the injection volume was kept at 20μl. A gradient elution was made by varying the proportion of solvent A to solvent B. The gradient elusion was 10% solvent A and 90% solvent B with flow rate 1 ml/min to 0.7 ml/min in 27min, from 10% to 40% solvent A, with flow rate 0.7 ml/min for 23min, 40% solvent A and 60% solvent B with flow rate 0.7 ml/min initially for 2min and afterward flow rate changed from 0.7 to 0.3 ml/min in 65min, from 40 to 44% solvent A with flow rate 0.3–0.7 ml/min in 70min, 44% solvent A with flow rate 0.7–1 ml/min for 10min duration, solvent A changed from 44% to 58% with flow rate 1 ml/min for 5min, 58–70% solvent A in 98 min at constant flow rate 1 ml/min. The versatile stage organization back to introductory condition (solvent A: solvent B: 10: 90) in 101min and permitted to run for another 4min, before the injection of another sample. The complete investigation time per sample was 105min. Each compound was recognized by its retention time and by spiking with standards under similar conditions. The quantification of phenolic and polyphenolic compounds in the methanol extract of the plant were carried out by the measurement of the integrated peak area and the contents were calculated using the calibration curve by plotting peak area against concentration of the respective standard sample.

The article "Evaluation of antioxidant activities, toxicity studies and the DNA damage protective effect of various solvent extracts of Litsea cubeba fruits" was retracted in 2024. Reasons: suspected computer-generated content; unreliable results or conclusions.

### 2.4 Toxicity studies and DNA protective activities of *L. cubeba*

Haemolytic toxicity of the aqueous (aq.) extracts of *L. cubeba* were carried out following the method of Malagoli 2007 [10] by mixing the various concentrations (100,200,300,500 and 1000 μg/ml) of fruit extracts to 10% suspension of rat erythrocytes. Cytotoxicity study of the aq. extracts of fruits were evaluated out by 3-(4,5-Dimethylthiazol-2-yl)-2,5-Diphenyltetrazolium Bromide (MTT) assay on isolated goat liver cells utilizing the convention as portrayed by Mosmann 1983 [11]. The genotoxic potential and DNA protective activity of the concentrates were assessed by single-cell gel electrophoresis comet examine as depicted by Singh et al. 1988 [12].

The ethical clearance for performing experiments on rodents erythrocytes, was obtained from Institutional Animal Ethics Committee (Approval No.- 04/P/S/IAEC/2017), Serampore College, West Bengal, India accommodating the CPCSEA rules. Goat liver was obtained straight from neighbourhood abattoir and brought on ice inside 30 min of death.

### 2.5 Statistical analysis

All the experiments were done using triplicate samples. Experimental results were subjected to univariate analysis of variance (ANOVA), followed by Tukey test (*p* ≤ 0.05) using the statistical package for the social sciences (SPSS version 7.5).

## 3 Results and discussion

The extractive value, content of phenolic compounds, flavonoids, reducing power, radical scavenging activities, metal chelating activity and lipid peroxidation assay of *L. cubeba* in five different solvent fractions are exhibited in Table 1.

**Table 1:** Antioxidant properties of *L.cubeba* and effect of different solvent extraction system.

Plant extract	Extractive value	Total phenolic content (Gallic acid equivalent) mg/100 gm DPM	Total flavonoid content (Rutin equivalent) mg/100 gm DPM	Reducing power (ascorbic acid equivalent) mg/100 gm DPM	DPPH radical scavenging activity (% of inhibition)	ABTS radical scavenging activity (% of inhibition)	FRAP assay mg/100 gm DPM	Metal chelating activity (% of inhibition)	Lipid peroxidation assay (% of inhibition)
Benzene	3.50 ± 0.34^d^	42.96 ± 1.76^e^	58.31 ± 1.09^d^	60.83 ± 3.49^e^	6.18 ± 0.18^e^	34.65 ± 0.26^e^	0.45 ± 0.04^e^	8.23 ± 0.07^e^	6.14 ± 0.38^e^
Chloroform	6.0 ± 0.28^c^	325.38 ± 2.80^d^	133.17 ± 1.08^c^	144.16 ± 2.26^d^	10.84 ± 0.43^d^	45.69 ± 0.54^d^	3.71 ± 0.03^d^	14.65 ± 0.16^d^	10.45 ± 0.29^d^
Acetone	6.50 ± 0.64^c^	413.84 ± 3.34^c^	136.15 ± 1.02^c^	234.74 ± 4.37^c^	13.91 ± 0.66^c^	60.76 ± 1.04^c^	8.38 ± 0.06^c^	18.34 ± 0.55^c^	16.34 ± 0.55^c^
Methanol	13.0 ± 0.21^b^	1011.28 ± 6.35^a^	259.09 ± 1.04^a^	458.65 ± 5.83^a^	40.35 ± 0.37^a^	88.68 ± 0.56^a^	17.42 ± 0.11^a^	26.56 ± 1.08^a^	21.45 ± 0.26^a^
Water	17.50 ± 1.03^a^	608.33 ± 5.68^b^	187.15 ± 1.68^b^	274.77 ± 3.68^b^	24.16 ± 1.33^b^	65.77 ± 1.44^b^	11.55 ± 1.34^b^	21.38 ± 1.11^b^	18.46 ± 1.33^b^

Each value in the table was obtained by calculating the average of three experiments and data are presented as Mean ± Standard error of the mean (SEM).Statistical analysis were carried out by Tukeys test at 95% confidence level and statistical significance were accepted at the p < 0.05 level. The superscript letter a,b,c,d and e denotes the significant differences within same parameters of different extract of the plant.

DPM: Dry plant material.

### 3.1 Antioxidant activities of *L. cubeba*

In our present investigation, *L. cubeba* extracts were acquired by using water, methanol, acetone, chloroform and benzene. Extraction yields extended from 3.50 ± 0.34 % for benzene extract to 17.50 ± 1.03 % for water extract (Table 1). The yields of extraction by several solvents reduced in the following direction: water > methanol > acetone > chloroform > benzene displaying that water possesses a significant high amount of % yield contents. It tends to be seen that the extraction yield of water (17.50%) is higher than that of unadulterated methanol (13.0%) and pure acetone (6.50%). These outcomes demonstrate that water enhances extraction yield. This might be owing to the higher solvency of proteins and carbohydrates in water and methanol than in chloroform, acetone and benzene [2].

The article "Evaluation of antioxidant activities, toxicity studies and the DNA damage protective effect of various solvent extracts of Litsea cubeba fruits" was retracted in 2024. Reasons: suspected computer-generated content; unreliable results or conclusions.

In the present study for extracting phenolic compounds from *L. cubeba* fruits, the water, methanol, acetone and benzene were used. Table 1 represents the total phenolic compounds in fractions expressed as gallic acid equivalents (GAE), varied between 42.96 ± 1.76 mg and 1011.28 ± 6.35 mg/100g dry plant material (DPM). The methanolic extract exhibited the highest total phenolics content (1011.28 ± 6.35 mg GAE/100g DPM), whereas the contents obtained with benzene were much smaller (42.96 ± 1.76 mg GAE/100g DPM). The extracting solvents essentially (P < 0.05) influenced the deliberate polyphenolic content. It is outstanding that dissolvable extremity will assume a key job in expanding phenolic dissolvability and methanol was exceptionally powerful dissolvable for the extraction of polar antioxidant agents. Furthermore methanol can impede phenol oxidase and hence is sensible for extraction of polyphenols [13].

The substance of all out flavonoids communicated as rutin reciprocals, shifted from 58.31 ± 1.09 to 259.09 ± 1.04 mg as rutin proportionate/100g DPM. The flavonoids content in the plants under assessment was generally surprising in methanol (259.09 ± 1.04 mg/100g DPM) sought after by water, acetone, chloroform and benzene. This data is in congruity to earlier report of most noteworthy flavonoids content from methanol concentrate of wild edible results of Meghalaya [14]. The plants rich in flavonoid content could be a decent wellspring of cancer prevention agents that would expand the general cell reinforcement limit of a life form and secure it against lipid peroxidation [15].

The reducing property of different extract of *L. cubeba* is stated as mg ascorbic acid equivalent (AAE)/100g DPM and is represented in Table 1. The reducing property of the cell reinforcement depends on the ability of giving a hydrogen atom to the free radical and along these lines balancing out them and breaking the free radical chain [16]. The reducing property of the dissolvable concentrate of *L. cubeba* can be positioned as methanol > water > chloroform > benzene, as exhibited in Table 1. Comparable perception was made by Sultana et al. (2007) [17] on restorative plants where the methanol concentrate indicated greatest reducing property and furthermore contained the most extreme phenolic content.

The article "Evaluation of antioxidant activities, toxicity studies and the DNA damage protective effect of various solvent extracts of Litsea cubeba fruits" was retracted in 2024. Reasons: suspected computer-generated content; unreliable results or conclusions.

The radical scavenging activity using DPPH radical and ABTS radical of the plant under investigation are shown in Table 1 and expressed as percentage of inhibition of dry extract. The antioxidant limit was evaluated utilizing DPPH and ABTS examines of different concentrates. Most extreme DPPH radical scavenging action was seen with methanol (40.35 ± 0.37%) and the activity lowered with reducing polarity. The outcome of present investigation is as per the investigation by Sultana et al. 2007 [17] on restorative plants where methanol displayed most extreme DPPH radical searching movement over solvent of low polarity. Similar results were obtained using ABTS radical, however this plant exhibited more prominent activity against ABTS radical. As per Hagerman, the high molecular weight phenolics have more capacities to extinguish free radicals (ABTS.+) and their adequacy relies upon the molecular weight, the number of aromatic rings and nature of hydroxyl groups substitution than the particular functional groups [18]. Free radical (ABTS·+) scavenging activity of *L. cubeba* fruits concentrates may be because of the nearness of high molecular weight phenolics, for example, catechin, and rutin derivatives. The methanol concentrate of *L. cubeba* fruits display noteworthy radical searching limit rendering, their use in various sicknesses related with oxidative pressure.

The Ferric reducing antioxidant power (FRAP) is expressed as μ mole Trolox equivalent (TE)/100g DPM and is summarized in Table 1. The methanol extract of *L cubeba* showed promising FRAP (17.42 ± 0.11mg/100g DPM) activity and least was observed with the benzene extract. In this assay, the presence of antioxidants in the plant extract brings about the reduction of Fe^+3^ to Fe^+2^ and it reflects the antioxidant capability of the test sample. They are electron donor and can diminish the intermediates of lipid peroxidation forms [19]. The outcomes shows that FRAP for water and methanol concentrate of the plant under examination were very close. Most elevated FRAP is seen in methanol concentrates which can be credited to its high substance of phenolics in this extract.

The Metal chelating activity of plant is expressed as % inhibition of metal ions and represented in Table 1. The maximum chelating activity is observed in methanol extract (26.56 ± 1.08%) followed by water (21.38 ± 1.11%), acetone (18.34 ± 0.55 %) extract and least was observed with benzene extract of the plant under study. Metal ion can start lipid peroxidation and initiate a chain reaction that prompts the disintegrating of sustenance [20]. The catalysis of metal particles in like manner relates with etiology of malignant growth and joint torment [21].

The article "Evaluation of antioxidant activities, toxicity studies and the DNA damage protective effect of various solvent extracts of Litsea cubeba fruits" was retracted in 2024. Reasons: suspected computer-generated content; unreliable results or conclusions.

The Anti-lipid peroxidation analyse was completed using five different extracts of *L. cubeba* and is expressed as % inhibition of lipid peroxidation/100g DPM and is represented in Table 1. Lipid peroxidation inhibition ability of the plant extracts can be ranked as methanol > water > acetone > chloroform > benzene fraction. The outcomes unmistakably infer those peroxidation are reliant on the extremity of the dissolvable utilized for extraction.

### 3.2 Identity and quantity of phenolic acids and flavonoids in *L. cubeba* by HPLC

Since methanol concentrate of the plant indicated better cell reinforcement exercises when contrasted with other dissolvable concentrates, the quantity of phenolic and polyphenolic compounds in *L. cubeba* by HPLC were done with the methanol concentrate of the plant.

The HPLC approach was effectively utilized for the distinguishing proof and extent of phenolics and polyphenolic compounds like gallic acid, protocatechuic acid, gentisic acid, chlorogenic acid, p-hydroxy benzoic acid, vanillic acid, caffeic acid, syringic acid, *p*-coumaric acid, ferulic acid, sinapic acid, salicylic acid and ellagic acid, catechin, rutin, myricetin, quercetin, naringin, apigenin and kaempferol in the methanol concentrate of *L. cubeba*.

The quantity of all phenolic acids and flavonoids in this plant has been communicated as μg/100mg dry extract (DE) and information introduced in Table 2.

**Table 2:** Phenolic acids and flavonoids content in *L. cubeba* by HPLC.

Phenolic acids/Flavonoids	Amount (μg/100mg dry extract)	Phenolic acids/Flavonoids	Amount (μg/100mg dry extract)
Gallic acid	2.52 ± 0.08^p^	Sinapic acid	37.45 ± 0.35^j^
Protocatechuic acid	46.42 ± 0.21^i^	Salicylic acid	15.23 ± 0.23^m^
Gentisic acid	ND	Naringin	ND
*p*-Hydroxy benzoic acid	1.56 ± 0.11^p^	Rutin	0.56 ± 0.02^q^
Catechin	72.04 ± 0.03^g^	Ellagic acid	106.08 ± 0.11^e^
Chlorogenic acid	29.76 ± 0.22^k^	Myricetin	7.58 ± 0.23^o^
Vanillic acid	28.60 ± 0.23^l^	Quercetin	9.97 ± 0.04^n^
Caffeic acid	145.71 ± 0.26^b^	Naringenin	107.47 ± 0.22^d^
Syringic acid	125.93 ± 0.07^c^	Apigenin	28.30 ± 0.14^l^
*p*-Coumaric acid	99.08 ± 0.19^f^	Kaempferol	53.29 ± 0.12^h^
Ferulic acid	155.60 ± 0.29^a^		

Each value in the table was obtained by calculating the average of three experiments and data are presented as Mean ± Standard error of the mean (SEM).Statistical analysis were carried out by Tukeys test at 95% confidence level and statistical significance were accepted at the p < 0.05 level. The superscript letter denotes the significant differences within same parameters of different extract of the plant.

The article "Evaluation of antioxidant activities, toxicity studies and the DNA damage protective effect of various solvent extracts of Litsea cubeba fruits" was retracted in 2024. Reasons: suspected computer-generated content; unreliable results or conclusions.

The HPLC chromatogram of the methanol extracts of the fruits *L. cubeba* (Figure 1.) showed the occurrence of gallic acid (2.52 ± 0.08) protocatechuic acid (46.42 ± 0.21), p-hydroxy benzoic acid (1.56 ± 0.11) catechin (72.04 ± 0.03), chlorogenic acid (29.76 ± 0.22), vanillic acid (28.60 ± 0.23 gm), caffeic acid (145.71 ± 0.26), syringic acid (125.93 ± 0.07), *p*-coumaric acid (99.08 ± 0.19), ferulic acid (155.60 ± 0.29), sinapic acid (37.45 ± 0.35), salicylic acid (15.23 ± 0.23), rutin (0.56 ± 0.02), ellagic acid (106.08 ± 0.11), myricetin (7.58 ± 0.23), quercetin (9.97 ± 0.04), naringenin (107.47 ± 0.22), apigenin (28.30 ± 0.14) and kaempferol (53.29 ± 0.12).

**Figure 1:** HPLC chromatogram of the methanol extract of the fruits of *L. cubeba* showing phenolic acids and flavonoids.

The HPLC examination revealed the occurrence of gallic acid which stays in the plant either in the free state or as ester and goes about as a ground-breaking cancer prevention agent. The gallic acid substance (2.52 ± 0.08 μg/100mg DE) in the methanol concentrate of *L. cubeba* is comparable to some normal vegetables to that in like manner vegetable like chilli pepper (3.33 mg/g), lemon (2.03 mg/g), spinach (1.82 mg/g), onion bulb (1.55 mg/g), cabbage (0.49 mg/g) and so on [22]. The plant found to contain protocatechuic acid (46.42 ± 0.21 μg/100mg DE) which is helpful for the treatment of different oxidative pressure related illnesses, for example, neurodegenerative and hepatic maladies [23]. The presence of *p*-hydroxybenzoic acid in the plant likewise legitimizes its uses on liver ailments, including liver cirrhosis and liver malignancy [24]. The utilization of this plant containing chlorogenic acid (29.76 ± 0.22) may be mindful to diminish glucose levels and possibly apply an enemy of diabetic impact [25]. The methanol concentrate of *L. cubeba* was found to contain 72.04 ± 0.03 μg/100mg catechin demonstrates that this plant may add to its restorative and cell reinforcement properties [26]. HPLC examination demonstrated the nearness of vanillic acid (28.60 ± 0.23 μg/100mg) in the explored plant which may be related with the hepatoprotective movement [27]. The present investigation demonstrated that products of *L. cubeba* were found to contain a generally excellent measure of caffeic acid (145.71 ± 0.26 μg/100mg) which is practically identical with the equivalent in cauliflower (5.8 μg/100mg), carrot (9.0 μg/100mg), lettuce (157.0 μg/100mg) and potato (280.0 μg/100mg) [28]. The awesome measure of syringic acid (125.93 ± 0.07 μg/100mg DE) in the fruit extract is notable for its enemy of malignancy, hostile to proliferative, narcotic, decongestant and hepato-defensive activities [29]. *p*-coumaric acid has been measured in *L. cubeba* (99.08 ± 0.19 μg/100mg DE) which demonstrates its defensive incentive as sustenance. The ferulic acid which is one of the significant phenolics, is exceptionally identified (155.60 ± 0.29 μg/100mg DE) in the methanol concentrate of *L. cubeba* in our examination and standard admission of the vegetable prompts bring down the cholesterol level in serum and builds sperm reasonability [30]. A lot of sinapic acid (37.45 ± 0.35 μg/100mg DE) was recognized in the plant under scrutiny and utilization of this plant would be helpful for wellbeing advancement since it demonstrated cell reinforcement, against microbial, mitigating, anticancer, and hostile to tension movement [31]. Rutin is a polyphenolic compound with glycosidic linkage having natural impacts, for example, antidiabetic impact [32], anticancer activities [33] and can possibly be utilized as a helpful operator. Considerable measure of rutin in *L. cubeba* proposes their potential use as helpful operators and legitimizes the legends application. A huge sum (106.08 ± 0.11 μg/100mg DE) of ellagic acid was recognized in the plant under scrutiny and utilization of this plant would be valuable for antimutagenic, antimicrobial and cell reinforcement properties, and inhibitors of human immunodeficiency infection (HIV) [31]. The fruits of *L. cubeba* contain obvious measure of myricetin and can be used for its antidiabetic prospective [34]. An extensive level of quercetin (9.97 ± 0.04 μg/100mg DE), recognized in the plant under examination were tantamount to the equivalent in apple (2.1μg/100mg), lettuce (1.1 μg/100mg) and tomato (5.5 μg/100mg) [35]. The presence of apigenin in the methanol concentrate of *L. cubeba* (28.30 ± 0.14 μg/100mg DE) might be helpful to diminish the danger of cardiovascular infirmities, neurological disorders, mutagenesis [36]. The utilization of this plant containing kaempferol (53.29 ± 0.12 μg/100mg DE) accordingly presenting incalculable medical advantages through lessening scourge of cardio vascular maladies, malignancy, arteriosclerosis and so on [37].

The article "Evaluation of antioxidant activities, toxicity studies and the DNA damage protective effect of various solvent extracts of Litsea cubeba fruits" was retracted in 2024. Reasons: suspected computer-generated content; unreliable results or conclusions.

### 3.3 Toxicity studies and DNA protective effect of *L. cubeba* extract

The eventual outcomes of the poisonous quality examinations of palatable plants including the reasonableness of cells and level of DNA damage using buffer (negative control) and hydrogen peroxide (positive control) were shown in Table 3.

**Table 3:** Toxicity studies of *L. cubeba*.

Name of the plant	Concentration of the extract (μg/ml)	Haemolytic toxicity RBC cell viability (%)	Hepatotoxicity Hepatocytes cell viability (%)	Genotoxicity % tail DNA
*L. cubeba*	100	94.42 ± 0.54	98.11 ± 0.24	3.54 ± 0.12
	200	91.07 ± 0.31	97.08 ± 0.16	4.06 ± 0.35
	300	89.16 ± 0.24	95.34 ± 1.16	4.74 ± 0.55
	500	88.05 ± 0.33	93.24 ± 1.11	4.92 ± 0.68
	1000	86.11 ± 0.18	91.26 ± 0.65	5.14 ± 0.52
Negative control	0	100.88 ± 1.03	99.56 ± 0.56	5.68 ± 0.81
Positive control (H_2_O_2_)	50 μM	78.34 ± 1.14	74.28 ± 1.08	25.18 ± 1.06
	100 μM	67.54 ± 1.32	66.20 ± 1.11	55.46 ± 1.44
	200 μM	50.11 ± 1.05	41.25 ± 1.05	76.35 ± 1.48

Each value in the table was obtained by calculating the average of three experiments and data are presented as Mean ± Standard error of the mean (SEM).

*In vitro* haemolytic activities on rodent erythrocytes of various obsessions (100,200,300, 500 and 1000 μg/ml) isolates got from satisfactory bits of wild plant under investigation were performed. The 50.11% haemolysis was gotten using H_2_O_2_ (200μM) and 100.88% cell sensibility was seen with buffer (Figure 2). The haemolysis started by packs in red platelets was obsession subordinate yet all focuses exhibited lower haemolytic effect on rodent red platelet at all core interests. The attainability of the haemolytic cell was most outrageous (94.42 ± 0.54%) at the very least centralization of 100 μg/ml of the plant under scrutiny and the most decreased was seen (86.11 ± 0.18%) at the most surprising part of 1000 μg/ml (Figure 2).

**Figure 2:** Haemolytic toxicity of *L. cubeba* and H_2_O_2_ (positive control).

Hepatocytes were isolated from fresh goat liver and the effects of various centers (100,200,300,500 and 1000 μg/ml) of aq. focuses of *L. cubeba* were seen on the sensibility of hepatocytes cell. The researched fruits showed most raised appropriateness (98.11 ± 0.24%) of the hepatocytes cell at a most minimal centralization of 100 μg/ml and the least (91.26 ± 0.65%) was seen at most astounding fixation (Figure 3). The rate practicality of RBC and hepatocytes cell for the plant removes at all obsessions (100–1000 μg/ml) were particularly equal to the negative control however the rate sensibility of both RBC and hepatocytes cell using H_2_O_2_ (Positive control) at a concentration 200 μM were 50.11 ± 1.05% and 41.25 ± 1.05% individually (Table 3).

**Figure 3:** Cytotoxicity of *L. cubeba* and H_2_O_2_ (positive control).

The genotoxicity examinations of plants incorporated the incubation of rodent lymphocytes in a low-melting point agarose (LMPA) suspension close by plant concentrate of different center (100–1000 μg/ml) followed by lysis of the cells in alkaline (pH > 13) conditions, and the electrophoresis of the suspended lysed cells. This was trailed by brief photographic examination of the slides with staining under Fluorescence microscope and registering fluorescence to choose the level of DNA damage. Olive Tail Moment (OTM) of individual stained nuclei was resolved using comet test programming. Negative control (whole blood and RPMI-1640) and positive controls (whole blood, 50, 100 and 200 μM H_2_O_2_ and RPMI-1640), were incorporated. A higher rate tail DNA exhibited an increasingly raised measure of DNA damage and progressively raised measure of genotoxicity of plant separate. The single cell gel electrophoresis inspect (comet test) is a modest, fundamental, and speedy method for assessing DNA strand breaks and in light of its affectability licenses examination at the individual cell level and the use of little models [8].

The article "Evaluation of antioxidant activities, toxicity studies and the DNA damage protective effect of various solvent extracts of Litsea cubeba fruits" was retracted in 2024. Reasons: suspected computer-generated content; unreliable results or conclusions.

The outcome of comet measure exhibited that the aq. extract of *L. cubeba* at a fixation 1000 μg/ml had the most raised rate (5.14 ± 0.52%) of tail DNA while the least rate (3.54 ± 0.12%) was found at 1000 μg/ml focus. The 5.68 ± 0.81% of tail DNA was obtained using negative control and positive control (mixture of entire blood, RPMI 1640 and 200 μM H_2_O_2_) demonstrated 76.35 ± 1.48% of tail DNA (Figure 4). The arrangement of free radicals during common assimilation causes mutagenicity and genotoxicity. In view of oxidative weight hydrogen peroxide showed part subordinate DNA hurt (25.18–76.35% of tail DNA) which was perceived by comet test. The outcome of assessment revealed that the level of DNA damage achieved by the plant evacuate at different obsessions were particularly similar to the negative control. Regular mixes, especially got from dietary sources give innumerable malignancy anticipation operators. Continuous examinations in individuals have shown that supplementation with cell support blends, for instance, nutrient E and C, lycopene and ß-carotene can help decrease levels of free-radical mischief apply a guarded effect against degenerative issue, for instance, dangerous development, by a decrease in DNA harm [38]. Plants have wide extent of pharmacologically convincing phytochemicals. A significant part of them have been represented steady for the treatment of a couple of afflictions of individual, yet couple of phytochemicals like saponin, tannin, cyanogenic glycosides, etc produce ruinous effects after introduction and can go about as ace oxidants, incorporate in all probability responsible for the mutagenicity and genotoxicity [39].

**Figure 4:** Genotoxicity of *L. cubeba* and H_2_O_2_ (positive control).

In the present investigation, the DNA defensive impact of the fluid concentrates of *L. cubeba* within the sight of 100 μM H_2_O_2_ (Figure 5), were then analyzed. The 55.46% of tail DNA was distinguished using H_2_O_2_ (positive control at a grouping of 100 μM). The watery concentrate of *L. cubeba* at 100,200,300, 500 and 1000 μg/ml showed a critical inhibitory impact on H_2_O_2_-prompted DNA harm (rate tail DNA 51.38, 46.24, 41.64, 33.08 and 26.18% individually). Hydrogen peroxide is a genotoxic operator, however it doesn't respond straightforwardly with DNA. Besides, within the sight of change metal particles, hydrogen peroxide delivers exceptionally responsive hydroxyl radicals through the Fenton response [40].

The article "Evaluation of antioxidant activities, toxicity studies and the DNA damage protective effect of various solvent extracts of Litsea cubeba fruits" was retracted in 2024. Reasons: suspected computer-generated content; unreliable results or conclusions.

**Figure 5:** DNA Protective effects of *L. cubeba*.

In the present exploration, because of acceptance of oxidative pressure, hydrogen peroxide delivered different degrees of harm to the DNA of isolated blood lymphocytes, which was recognized by the comet measure. We found that all groupings of hydrogen peroxide (50, 100, and 200 μM) caused portion ward harm to DNA of lymphocytes. We likewise found that fluid concentrates of *L. cubeba* caused DNA harm in rodent lymphocytes to lesser degree (Table 3). The watery concentrate of *L. cubeba* showed defensive exercises against H_2_O_2_-incited chromosomal harm. The antioxidant activities and HPLC examination of *L. cubeba* recommended to be identified with the constituents, for example, rutin, myricetin kaempferol, quercetin, apigenin which can search free radicals and block the peroxidation of nucleic acids and DNA harm, just as diminish the creation of free radicals [8]. Considering the constituents present in the fluid *L. cubeba* separate, our information propose that fluid concentrate of the plant under scrutiny has defensive impacts against hydrogen peroxide-instigated oxidative DNA harm in rodent lymphocytes. Consequently, *L. cubeba* may have potential for the counteractive action and treatment of sicknesses coming about because of oxidative stress.

## 4 Conclusion

The result of present examination showed the presence high phenolics and flavonoids in the aqueous extract of *L. cubeba* fruits which also reflected in the observed free radical scavenging, reducing and iron-chelating capacity of this extract.

The results of haemolytic toxicity, cytotoxicity and genotoxicity of this edible plant revealed that this is non-toxic at cell and genomic level and safe to consume. The aqueous extract of the fruit possessing DNA protective activity against hydrogen peroxide initiated oxidative DNA harm in rodent lymphocytes. So we acknowledge that this fruit could be used for the stimulating explanation behind individual as a result of their incredible feeding qualities, and adequate security may be gotten against illnesses rising up out of absence of solid sustenance. The preliminary disclosures moreover revealed that this wild consumable fruit was the incredible wellspring of enhancement for intrinsic masses. Therefore, the advancement of this wild palatable fruits ought to be grasped in colossal scale, which will convey monetary focal points for underprivileged farmers.

The article "Evaluation of antioxidant activities, toxicity studies and the DNA damage protective effect of various solvent extracts of Litsea cubeba fruits" was retracted in 2024. Reasons: suspected computer-generated content; unreliable results or conclusions.

## Declarations

### Author contribution statement

Tapan Seal: Conceived and designed the experiments; Performed the experiments; Analyzed and interpreted the data; Contributed reagents, materials, analysis tools or data; Wrote the paper.

Kausik Chaudhuri, Basundhara Pillai, Tanmoy Mondal: Performed the experiments.

Shrabana Chakrabarti: Conceived and designed the experiments; Performed the experiments; Analyzed and interpreted the data.

Biswajit Auddy: Analyzed and interpreted the data.

### Funding statement

This research did not receive any specific grant from funding agencies in the public, commercial, or not-for-profit sectors.

### Competing interest statement

The authors declare no conflict of interest.

### Additional information

No additional information is available for this paper.
